RETRACTED

# Cucurbitacin E inhibits osteosarcoma cells proliferation and invasion through attenuation of PI3K/AKT/mTOR signalling pathway

**DOI:** 10.1042/BSR20160165

**Published:** 2016-11-08

**Authors:** Ying Wang, Shumei Xu, Yaochi Wu, Junfeng Zhang

**Affiliations:** * Department of Acupuncture, Tuina and Traumatology, the Sixth People's Hospital Affiliated to Shanghai Jiaotong University, Shanghai 200233, China; † Department of Hepatobiliary Surgery, Lanzhou General Hospital, Lanzhou Command of CPLA, Lanzhou 730050, China

**Keywords:** apoptosis, cell cycle, cucurbitacin E, osteosarcoma, PI3K, Akt, mTOR signalling, proliferation

## Abstract

Cucurbitacin E (CuE), a potent member of triterpenoid family isolated from plants, has been confirmed as an antitumour agent by inhibiting proliferation, migration and metastasis in diverse cancer. However, the effects and mechanisms of CuE on osteosarcoma (OS) have not been well understood. The present study aimed to test whether CuE could inhibit growth and invasion of OS cells and reveal its underlying molecular mechanism. After various concentrations of CuE treatment, the anti-proliferative effect of CuE was assessed using the cell counting Kit-8 assay. Flow cytometry analysis was employed to measure apoptosis of OS cells. Cell cycle distribution was analysed by propidium iodide staining. Transwell assay was performed to evaluate the effect of CuE on invasion potential of OS cells. The protein levels were measured by western blot. In addition, the potency of CuE on OS cells growth inhibition was assessed *in vivo*. Our results showed that CuE inhibited cell growth and invasion, induced a cell cycle arrest and triggered apoptosis and modulated the expression of cell growth, cell cycle and cell apoptosis regulators. Moreover, CuE inhibited the PI3K/Akt/mTOR pathway and epithelial–mesenchymal transition (EMT), which suppressed the invasion and metastasis of OS. In addition, we also found that CuE inhibited OS cell growth *in vivo*. Taken together, our study demonstrated that CuE could inhibit OS tumour growth and invasion through inhibiting the PI3K/Akt/mTOR signalling pathway. Our findings suggest that CuE can be considered to be a promising anti-cancer agent for OS.

## INTRODUCTION

Osteosarcoma (OS) is the most prevalent primary malignant bone tumour and the leading cause for cancer-related death among children and adolescents [1]. Although the 5-year survival of patients with localized OS has improved to 60–80% due to the multi-agent, dose-intensive chemotherapy in conjunction with gradually improved surgical techniques, prognosis remains unsatisfactory [2]. At the same time, the high-dose use of chemotherapeutic drugs (methotrexate, doxorubicin, cisplatin and ifosfamide) is limited due to their systemic toxicity, such as nephrotoxicity and neurotoxicity [3–6]. Therefore, the development of novel therapies for the management of OS is especially urgent.

RETRACTED

Increasing evidence supports that natural agents open up a novel avenue for treatment of cancers, especially by combining with conventional therapeutics [7]. Cucurbitacin E (CuE), a natural tetracyclic triterpenoid, is an abundant member of the cucurbitacin family, which is widely distributed in the plants [8]. It has been well documented that cucurbitacins inhibit growth and proliferation in various cancer cells via cell cycle arrest, and induction of apoptosis [9]. Recent observations showed that CuE also suppressed the proliferation and induced apoptosis in ovarian [10,11], leukaemia [12] and pancreatic cancer cell lines [13]. However, limited studies have paid attention on the therapeutic effects and underlying mechanisms of CuE on OS.

PI3K/Akt/mTOR pathway is a major signalling cascade which operates downstream to the receptor tyrosine kinases such as epidermal growth factor receptor (EGFR), platelet-derived growth factor receptor (PDGFR) and insulin-like growth factor-1 receptor (IGF-1R) [14,15]. Recent researches support that PI3K/Akt/mTOR pathway play indispensable roles in many biological processes such as the cell proliferation, survival, migration, angiogenesis and metabolism in breast cancer, bladder cancer and so on [16–19]. Song et al. found that P53 suppressed cell proliferation and angiogenesis of OS through inhibition of the PI3K/AKT/mTOR pathway [20]. However, whether the PI3K/Akt/mTOR pathway participates in the anticancer effects of CuE is unknown.

In the present study, the effects and underlying molecular mechanisms of the anticancer action of CuE were explored in MG63 and U2OS cells. The results suggested that CuE could suppress OS cells proliferation and invasion, induce G2/M cell cycle arrest and trigger apoptosis *in vitro*. Moreover, CuE blocked PI3K/Akt/mTOR pathway and inhibited EMT in OS cells. In addition, CuE could also inhibit MG63 and U2OS cells *in vivo* growth. In conclusion, our data showed CuE inhibited OS cells proliferation and invasion through attenuation of PI3K/AKT/mTOR signalling.

## MATERIALS AND METHODS

### Cells and regents

Human OS cell line MG63 and U2OS were obtained from A.T.C.C. All cell lines were carefully incubated at 37°C under a humidified 5% CO_2_. CuE (MF: C_32_H_44_O_8_, MW: 540.7, purity>98%) was purchased from the Department of Pharmacy, Shenyang Pharmaceutical University, China and dissolved using the solvent system: chloroform/methanol (9:1). Antibodies of PCNA, Ki-67, Cyclin B1, CDC2 and phospho-CDC2 (Tyr^15^) were purchased from Cell Signaling, and antibodies of Caspase-3, Caspase-8, Bcl-2, ZEB1, E-cadherin, N-cadherin, vimentin, p-Akt, Akt, p-mTOR, mTOR and β-actin were purchased from Santa Cruz. Anti-rabbit IgG and anti-mouse IgG were used as secondary antibodies (Santa Cruz Biotechnology).

RETRACTED

### Cell culture and treatments

Human OS cell line MG63 and U2OS cultured in Dulbecco's modified Eagle medium (DMEM; Invitrogen Gibco Cell Culture Products) supplemented with 10% FBS (Invitrogen) at 37°C in a humidified atmosphere of 95% air and 5% CO_2_. The cells treated with CuE (0, 1 and 2.5 μM) were collected at 72 h for further measurements.

### Cell viability assay

MG63 and U2OS cells were seeded in 96-well culture plates with 1×10^4^ cells/well, and incubated at 37°C with 5% CO_2_. After treating with different concentrations (0, 0.01, 0.1, 1, 2.5, 5 and 10 μM) of CuE, the cell viability assay was performed using Cell Counting Kit-8 (CCK-8; Dojindo) according to the manufacturer's protocol. The absorbance at 450 nm was measured.

### Cell apoptosis detection by flow cytometry

MG63 and U2OS cells were collected after treatment with the indicated concentrations of CuE (0 and 2.5 μM), and then washed twice with PBS. Apoptotic cells were measured with an Annexin V-FITC/PI detection kit (Invitrogen Life Technologies). The cells were resuspended in 500 μl binding buffer at a concentration of 10^6^/ml and then mixed with 10 μl Annexin V (Bio-Science) for 10 min in the dark at room temperature (RT), followed by the addition of 5 μl PI (Bio-Science). After incubation at RT in the dark for 5 min, samples were analysed by an Epics Altra Flow Cytometer (Beckman Coulter).

### Cell cycle analysis

Cells (1×10^6^) were incubated with the indicated concentrations of CuE (0 and 2.5 μM) for adequate time, collected by gentle trypsinization and re-suspended in PBS. After fixation in 70% cold ethanol at −20°C for at least 1.5 h, cells were stained with PI-working solution (40 μg/ml PI and 100 μg/ml RNase A and 0.1% Triton X-100) at 37°C for 1 h and then analysed for cell cycle distribution by flow cytometry. Flow cytometry was carried out on an Epics Altra Flow Cytometer and was analysed using EXPO32 Multicomp and EXPO32 v1.2 Analysis (Beckman Coulter) software.

### Invasion assay

The Transwell assay was performed as described before [21]. Briefly, the upper surface of the transwell membrane were coated with 20 μl Matrigel and the lower compartment of the chambers were filled with 500 μl medium containing 10% FBS. 1.25 ×10^5^ cells in 100 μl serum-free medium were placed in the upper part of each transwell and treated with the indicated concentrations of CuE (0 and 2.5 μM). After incubation for 24 h, cells on the upper side of the filter were removed. Cells located on the underside of the filter were fixed with 4% paraformaldehyde and stained with Giemsa solution and counted in five randomly selected fields under a microscope. Percentage inhibition of migratory cells was quantified.

RETRACTED

### Tumour xenograft animal model

Male athymic nude mice were housed and manipulated according to the protocols approved by the Shanghai Medical Experimental Animal Care Commission. Animal experiments were conducted in accordance with the guidelines of Shanghai Jiaotong University and the National Institutes of Health (NIH). For each mouse, MG63 and U2OS cells (five million cells in 0.1 ml of culture medium) were subcutaneously injected at the right thigh of nude mice, and treatment was started when the tumours reached an average volume of 200–300 mm^3^. All mice were divided into three groups (*n*=10 in each group). CuE (0, 1.0 and 5.00 mg/kg per 2 days) or DMSO was given via intraperitoneal injection. Mice tumour weight (at week 5) was recorded. The tumour volume (in mm^3^) was calculated by the formula: volume=(width)^2^×length/2, and the tumour growth curve was presented.

### Western blot

After treatment with different concentrations of CuE (0, 1 and 2.5 μM) for 24 h, cells were washed twice with cold PBS and harvested using cell scrapes and quantified by BCA method. Equal amounts of protein extracts were loaded on to SDS/PAGE and ran at 100 mV for 80 min, followed by transferring to PVDF membranes at 100 mV for 30 min at room temperature. The membrane was blocked in 5% non-fat milk, and then incubated with primary antibodies as indicated. Subsequent to being incubated with anti-rabbit or anti-mouse secondary antibodies (Santa Cruz Biotechnology) for 1 h, the immune complexes were detected using the enhanced chemiluminescence (ECL) method. Blot intensity was quantified though the Image J software.

### Statistical analysis

All values are expressed as mean±standard deviation (S.D.) and performed in triplicate. One Way ANOVA was used to compare the difference between control and concentration treatments in each group followed by Bonferroni's multiple comparison tests. A *P* value of less than 0.05 was considered to be statistically significant.

## RESULTS

### CuE induces cytotoxic effect in cultured OS cells

First, we tested the potential cytotoxicity of CuE against OS cells. After 24 h treatment, two OS (MG63 and U2OS) cells viability in the presence of concentrations of 0.01, 0.1, 1, 2.5, 5 and 10 μM CuE was significantly inhibited compared with that of controls (0 μM) in CCK-8 assay (Figures 1A and 1B). Previous studies have addressed that PCNA and Ki-67 were excellent markers for determining the growth cell fraction of a given cell population [22]. Hence, we observed the expression of PCNA and Ki-67 in OS cells. As shown in Figures 1(C) and 1(D), CuE decreased the expression of PCNA and Ki-67 in a dose-dependent manner. These results together show that CuE treatment induces cytotoxic effect against OS cells.

RETRACTED

**Figure 1:** CuE inhibited cell survival of MG63 and U2OS cells (**A**–**B**) Cell proliferation activity was measured by CCK-8 assays in MG63 (**A**) and U2OS (**B**) cells. Cells were treated with various concentrations of CuE as indicated. (**C**–**D**) The expressions of Ki-67 and PCNA were detected in MG63 (**C**) and U2OS (**D**) cells by western blot. All data were reported as the mean±S.E.M. of at least three separate experiments. **P<0.01 compared with untreated group.

### CuE blocks G2/M phase cell cycle progression in MG63 and U2OS cells

To test whether CuE modulates the cell cycle among OS cells, we treated MG63 and U2OS cells with 2.5 μM CuE for 24 h, after which we measured cell cycle distribution. As shown in Figures 2(A)–2(D), ratio of G2/M increased dramatically in both MG63 and U2OS cells lines treated with CuE (2.5 μM) when compared with untreated group (0 μM). To gain further insight into the mechanism of CuE-induced cell cycle arrest at G2/M, we determined the expression of Cyclin B1, CDC2, as well as phospho-CDC2 at Tyr^15^ using WB. As shown in Figures 2(E) and 2(F), the expression of phospho-CDC2 at Tyr^15^ and Cyclin B1 decreased greatly in OS cells treated with CuE at different dosages (1 and 2.5 μM) when compared with untreated group. In contrast, no significant effects at different concentrations of 1 and 2.5 μM of CuE on CDC2 expression were noted in western blotting analysis. Thus, it appears that inactivation of phospho-CDC2 and down-regulation of Cyclin B1 may be involved in CuE-induced cell cycle arrest at G2/M.

**Figure 2:** CuE induces cell cycle G2/M arrest in MG63 and U2OS cells (**A** and **B**) MG63 and U2OS cells were treated with CuE (0 and 2.5 μM) for 24 h. Cells were stained with PI and analysed by flow cytometry. The cell cycle graph was analysed by FlowJo software (version 7.6). (**C** and **D**) CuE significantly increased the percentage of G2/M phase in MG63 and U2OS cells compared with untreated group. (**E** and **F**) MG63 and U2OS cells were treated with CuE (0, 1.0 and 2.5 μM) for 24 h respectively. Protein levels of Cyclin B1, CDC2 and phospho-CDC2 (Tyr^15^) were examined by western blot. Protein levels of β-actin were measured as loading controls. All data were reported as the mean±S.E.M. of at least three separate experiments. **P<0.01 compared with untreated group. See Supplementary Material for large format version of Figure 2.

RETRACTED

### CuE induces apoptosis in MG63 and U2OS cell lines

To detect whether the reduction in cell viability was associated with cell apoptosis, flow cytometry assay was applied to detect the apoptotic rate of MG63 and U2OS cells treated with CuE. As shown in Figures 3(A)–3(D), compared with untreated group, apoptosis was markedly increased in both MG63 and U2OS cells after treatment with 2.5 μM CuE for 48 h. After noting that CuE-induced apoptosis, we further examined the protein levels of apoptosis regulators using Western blot analysis. In both MG63 and U2OS cells, CuE (1 and 2.5 μM) treatment for 24 h significantly increased the expression of Caspase-3 and Caspase-8. Meanwhile, CuE administration dramatically decreased the levels of anti-apoptotic protein, Bcl-2 (Figures 3E and 3F). These results suggest that the CuE could induce apoptosis in OS cells by caspase-dependent process.

**Figure 3:** CuE induces apoptosis in MG63 and U2OS cells MG63 (**A**) and U2OS (**B**) cells were treated with CuE (0 and 2.5 μM) for 24 h. Cells were stained with Annexin V/propidium iodide (PI), and apoptosis was determined using flow cytometry. (**C**–**D**) Apoptosis rates of MG63 (**C**) and U2OS (**D**) cells with CuE (0 and 2.5 μM) treatment were represented. (**E** and **F**) Protein levels of Caspase-3, Caspase-8 and Bcl-2 were examined by western blot. MG63 (**E**) and U2OS (**F**) cells were treated with CuE (0, 1.0 and 2.5 μM) for 48 h respectively. Protein levels of β-actin were measured as loading controls. All data were reported as the mean±S.E.M. of at least three separate experiments. **P<0.01 compared with untreated group.

### CuE inhibits the invasion of MG63 and U2OS cells

It has reported that CuE blocked breast cancer metastasis by suppressing tumour cell migration and invasion [23]. To further understand the biological functions of CuE in OS cell migration and invasion, we treated both MG63 and U2OS cells with 2.5 μM CuE. As expected, we found that CuE significantly inhibited the invasion of MG63 and U2OS cells compared with untreated group (Figures 4A–4D). Because epithelial-to-mesenchymal transition (EMT) plays a critical role in invasion and metastasis of OS [24] and cucurbitacin B (CuB), a close analogue of CuE, mediated HER2/TGFβ inhibition lead to suppression of EMT in breast cancer cells [25]. Hence, we observed the expression of EMT related genes in OS cells. The low level of EMT was confirmed by the decrease in mesenchymal marker N-cadherin and vimentin in both MG63 and U2OS cells along with promotion of epithelial markers E-cadherin and ZEB1 (Figures 4E and 4F). These observations suggest that CuE inhibits OS cells invasion through regulating EMT process.

RETRACTED

**Figure 4:** CuE inhibits invasion in MG63 and U2OS cells **(A** and **B**) CuE inhibits MG63 and U2OS invasion. Tumour cells were treated with different concentrations of CuE and allowed to invade through Matrigel. (**C** and **D**) Invaded cell number was counted. (**E** and **F**) Protein levels of ZEB1, E-cadherin, vimentin and N-cadherin were examined by western blot. MG63 (**E**) and U2OS (**F**) cells were treated with CuE (0, 1.0 and 2.5 μM) after 24-h incubation. Protein levels of β-actin were measured as loading controls. All data were reported as the mean±S.E.M. of at least three separate experiments. **P<0.01 compared with untreated group.

### CuE inhibits PI3K/Akt/mTOR-signalling pathway

Recent studies demonstrated that aberration of PI3K/Akt/mTOR pathway is a very common mechanism for many human cancers including OS, since it can mediate survival pathway and apoptosis pathway [26]. A growing number of studies revealed that inhibition of PI3K/Akt pathway, using grifolin, could induce apoptosis of human OS cells [27]. Therefore, we investigated the effects of CuE on the PI3K/Akt/mTOR-signalling pathway in MG63 and U2OS cells. As shown in Figures 5(A)–5(D), the protein expression levels of p-AKT, p-p70S6K and p-mTOR were significantly down-regulated, whereas the expression levels of p-4EBP1 was up-regulated in a dose-dependent manner in both MG63 and U2OS cells. These dates indicated that CuE could inhibit tumour growth by blocking the PI3K/Akt/mTOR-signalling pathway.

**Figure 5:** CuE alters the expression of key components in the PI3K/Akt pathway (**A** and **B**) Expression changes of the Akt, mTOR, p70S6K and 4EBP1 genes at the translational level in CuE-treated MG63 cells. (**C** and **D**) Western blotting analysis of relative protein expression in CuE-treated or non-treated U2OS cells. CuE significantly inhibited the expression of Akt, mTOR and p70S6K protein, but increased the expression of 4EBP1 protein. All data were reported as the mean±S.E.M. of at least three separate experiments. **P<0.01 compared with untreated group.

### CuE inhibits tumorigenesis in OS cells *in vivo*

To further investigate the inhibitory function of CuE on OS metastasis *in vivo*, MG63 and U2OS cells were subcutaneously injected at the right thigh of nude mice, and treated it with different concentrations CuE (1.0 and 5.0 mg/kg). As a result, we found that the average tumour volume and weight in mice treated with MG63 injection were significantly reduced compared with untreated group after CuE treatment (Figures 6A, 6C and 6E). Moreover, similar results were also obtained in mice treated with U2OS injection (Figures 6B, 6D and 6F). This result further confirmed that CuE was a potential agent for inhibiting tumorigenesis.

RETRACTED

**Figure 6:** CuE inhibits MG63 and U2OS cell growth in tumour xenograft mice model MG63 and U2OS cells (five million cells in 0.1 ml of culture medium) were subcutaneously injected at the right thigh of nude mice, and treatment was started when the tumours reached an average volume of 200–300 mm^3^. Animals were randomized into three groups with 20 mice each group: (**a**) 0 mg/kg of CuE; (**b**) 1.0 mg/kg of CuE; (**c**) 5.0 mg/kg of CuE. CuE was injected intraperitoneally (i.p.) twice daily for 1 week. (**A** and **B**) Tumour volume (in mm^3^, recorded every week). (**C** and **D**) Tumour weight (in grams, recorded every week). Data were expressed as mean±S.D., experiments were repeated three times. (**E** and **F**) CuE significantly inhibited the tumour formation of MG63 and U2OS cells in a nude mouse xenograft model. *P<0.05, **P<0.01 compared with untreated group.

## DISCUSSION

In present study, we proved the roles and molecular mechanisms of CuE in OS cells. The antitumour activity of CuE was demonstrated *in vitro* and in animal models. Furthermore, our results showed that CuE inhibited the PI3K/Akt/mTOR pathway along with the suppression of the phosphorylation of PI3K downstream factors including AKT, mTOR and P70S6K. These results show that CuE suppresses cell proliferation and invasion of OS through inhibition of the PI3K/AKT/mTOR pathway, which might be an effective novel therapeutic candidate against OS in the future.

Several reports have demonstrated that cucurbitacins exhibited a wide range of biological activities, such as anti-inflammatory [28], anti-fertility [8] and anti-cancer [29]. CuE (a-elaterin), one of cucurbitacins, could disrupt cell actin filaments and inhibit cell adhesion [30]. More evidences have found that CuE inhibited cell proliferation and induced cell cycle arrest at G2/M phase in several different cancer cell lines [31,32]. And, a study from Zhang et al. [23] showed that CuE inhibited tumour cell migration by impairing Arp2/3-dependent actin polymerization in breast cancer, which indicated the potential therapeutic effects of CuE on prostate cancer. However, little attention has been paid to the effects of CuE in OS. In the present study, we demonstrated that CuE inhibited cell growth in OS cell lines in a dose-dependent manner. To elucidate the effect of CuE on the growth of OS cells, we have performed a series of experiments on cell cycle distribution and apoptosis. The results showed that CuE induced a cell cycle arrest and triggered apoptosis and modulated the expression of cell growth, cell cycle and cell apoptosis regulators. Therefore, the inhibitory effect of CuE on OS cell growth may be due to induction of cell cycle arrest as well as apoptosis. In addition, our vitro results demonstrated that CuE inhibited the invasion of OS cells by suppression of EMT and our vivo results showed that administration of CuE decreased tumour growth in a dose-dependent manner, which indicated that CuE has potential as an inhibitor of OS metastasis.

RETRACTED

Increasing studies have demonstrated that PI3K/AKT/mTOR signalling pathway participated in the progression of kinds of cancers including OS. For example, Yang et al. [33] found that XBP1 exerted its effect on OS probably by influencing PI3K/mTOR signalling. A study performed by Liu et al. [34] showed that lupeol can induce apoptosis as well as cell cycle arrest of human OS cells through phosphatidylinositol 3-kinase/AKT/mammalian target of rapamycin pathway. However, it is unknown whether PI3K/AKT/mTOR signalling pathway mediated the anti-cancer effect of CuE. Recently, Jia et al. [35] reported that CuE exerted its anti-inflammatory properties in human synoviocyte MH7A cells via modulation of PI3K/Akt/NF-κB pathway. In the present study, to understand the mechanism by which CuE can lead to cell growth, we have measured p-AKT, p-p70S6K, p-mTOR and p-4EBP1. Our data showed that CuE treatment decreased the protein expression levels of p-AKT, p-p70S6K, p-mTOR, whereas promoted the expression levels of p-4EBP1, indicating that CuE may be an important regulator of this signalling pathway. These data indicate that CuE may exert its anti-cancer effect by regulating the PI3K/Akt/mTOR-signalling pathway.

In conclusion, our data demonstrated that CuE inhibited OS cells proliferation and invasion, at least, partially through attenuation of PI3K/AKT/mTOR signalling pathway in OS. The ability of CuE to inhibit OS cell growth may provide a new and potential therapeutic agent for the OS treatment. However, emerging reports showed that other pathways also contribute to the initiation and progression of OS. Therefore, examining the roles of other pathways in CuE-induced growth inhibition in OS cells warrants our future research.

## Abbreviations

CCK-8: Cell Counting Kit-8
CuE: cucurbitacin E
EGFR: epidermal growth factor receptor
EMT: epithelial–mesenchymal transition
IGF-1R: insulin-like growth factor-1 receptor
OS: osteosarcoma
PDGFR: platelet-derived growth factor receptor
RT: room temperature

## References

[1] Picci P. (2007). Osteosarcoma (osteogenic sarcoma). Orphanet. J. Rare Dis..

RETRACTED

[2] Jaffe N. (2009). Osteosarcoma: review of the past, impact on the future. The American experience. Cancer Treat. Res..

[3] Bailey D., Erb H., Williams L., Ruslander D., Hauck M. (2003). Carboplatin and doxorubicin combination chemotherapy for the treatment of appendicular osteosarcoma in the dog. J. Vet. Intern. Med..

[4] Ferguson W.S., Harris M.B., Goorin A.M, Gebhardt M.C., Link M.P., Shochat S.J., Siegal G.P., Devidas M., Grier H.E. (2001). Presurgical window of carboplatin and surgery and multidrug chemotherapy for the treatment of newly diagnosed metastatic or unresectable osteosarcoma: Pediatric Oncology Group Trial. J. Pediatr. Hematol. Oncol..

[5] Muggia F.M., Louie A.C. (1978). Five years of adjuvant treatment of osteosarcoma: more questions than answers. Cancer Treat. Rep..

[6] Carter S.K. (1984). Adjuvant chemotherapy in osteogenic sarcoma: the triumph that isn't?. J. Clin. Oncol..

[7] Li Y., Kong D., Wang Z., Sarkar F.H. (2010). Regulation of microRNAs by natural agents: an emerging field in chemoprevention and chemotherapy research. Pharm. Res..

[8] Chen J.C., Chiu M.H., Nie R.L., Cordell G.A., Qiu S.X. (2005). Cucurbitacins and cucurbitane glycosides: structures and biological activities. Nat. Prod. Rep..

[9] Chen X., Bao J., Guo J., Ding Q., Lu J., Huang M., Wang Y. (2012). Biological activities and potential molecular targets of cucurbitacins: a focus on cancer. Anticancer Drugs.

[10] Shan X.L., Zhou X.Y., Yang J., Wang Y.L., Deng Y.H., Zhang M.X. (2010). [Inhibitory effect of cucurbitacin E on the proliferation of ovarian cancer cells and its mechanism]. Chin. J. Cancer.

[11] Sadzuka Y., Hatakeyama H., Sonobe T. (2010). Enhancement of doxorubicin concentration in the M5076 ovarian sarcoma cells by cucurbitacin E co-treatment. Int. J. Pharm..

[12] Li Y., Wang R., Ma E., Deng Y., Wang X., Xiao J., Jing Y. (2010). The induction of G2/M cell-cycle arrest and apoptosis by cucurbitacin E is associated with increased phosphorylation of eIF2alpha in leukemia cells. Anticancer Drugs.

[13] Sun C., Zhang M., Shan X., Zhou X., Yang J., Wang Y., Li-Ling J., Deng Y. (2010). Inhibitory effect of cucurbitacin E on pancreatic cancer cells growth via STAT3 signaling. J. Cancer Res. Clin. Oncol..

[14] Ludwig J.A., Lamhamedi-Cherradi S.E., Lee H.Y., Naing A., Benjamin R. (2011). Dual targeting of the insulin-like growth factor and collateral pathways in cancer: combating drug resistance. Cancers (Basel).

[15] Arcaro A., Guerreiro A.S. (2007). The phosphoinositide 3-kinase pathway in human cancer: genetic alterations and therapeutic implications. Curr. Genomics.

[16] Yap T.A., Garrett M.D., Walton M.I., Raynaud F., de Bono J.S., Workman P. (2008). Targeting the PI3K-AKT-mTOR pathway: progress, pitfalls, and promises. Curr. Opin. Pharmacol..

RETRACTED

[17] McAuliffe P.F., Meric-Bernstam F., Mills G.B., Gonzalez-Angulo A.M. (2010). Deciphering the role of PI3K/Akt/mTOR pathway in breast cancer biology and pathogenesis. Clin. Breast Cancer.

[18] Ching C.B., Hansel D.E. (2010). Expanding therapeutic targets in bladder cancer: the PI3K/Akt/mTOR pathway. Lab. Invest..

[19] Liu P., Cheng H., Roberts T.M., Zhao J.J. (2009). Targeting the phosphoinositide 3-kinase pathway in cancer. Nat. Rev. Drug Discov..

[20] Song R., Tian K., Wang W., Wang L. (2015). P53 suppresses cell proliferation, metastasis, and angiogenesis of osteosarcoma through inhibition of the PI3K/AKT/mTOR pathway. Int. J. Surg..

[21] Pan X., Han H., Wang L., Yang L., Li R., Li Z., Liu J., Zhao Q., Qian M., Liu M., Du B. (2011). Nitidine chloride inhibits breast cancer cells migration and invasion by suppressing c-Src/FAK associated signaling pathway. Cancer Lett.

[22] Mambelli L.I., Mattos R.C., Winter G.H., Madeiro D.S., Morais B.P., Malschitzky E., Miglino M.A., Kerkis A., Kerkis I. (2014). Changes in expression pattern of selected endometrial proteins following mesenchymal stem cells infusion in mares with endometrosis. PLoS One.

[23] Zhang T., Li J., Dong Y., Zhai D., Lai L., Dai F., Deng H., Chen Y., Liu M., Yi Z. (2012). Cucurbitacin E inhibits breast tumor metastasis by suppressing cell migration and invasion. Breast Cancer Res. Treat..

[24] Cheng H.L., Lin C.W., Yang J.S., Hsieh M.J., Yang S.F., Lu K.H. (2016). Zoledronate blocks geranylgeranylation not farnesylation to suppress human osteosarcoma U2OS cells metastasis by EMT via Rho A activation and FAK-inhibited JNK and p38 pathways. Oncotarget.

[25] Gupta P., Srivastava S.K. (2014). HER2 mediated *de novo* production of TGFbeta leads to SNAIL driven epithelial-to-mesenchymal transition and metastasis of breast cancer. Mol. Oncol..

[26] Chen J., Yao D., Yuan H., Zhang S., Tian J., Guo W., Liang W., Li H., Zhang Y. (2013). Dipsacus asperoides polysaccharide induces apoptosis in osteosarcoma cells by modulating the PI3K/Akt pathway. Carbohydr. Polym..

[27] Jin S., Pang R.P., Shen J.N., Huang G., Wang J., Zhou J.G. (2007). Grifolin induces apoptosis via inhibition of PI3K/AKT signalling pathway in human osteosarcoma cells. Apoptosis.

[28] Qiao J., Xu L.H., He J., Ouyang D.Y., He X.H. (2013). Cucurbitacin E exhibits anti-inflammatory effect in RAW 264.7 cells via suppression of NF-kappaB nuclear translocation. Inflamm. Res..

[29] Jayaprakasam B., Seeram N.P., Nair M.G. (2003). Anticancer and antiinflammatory activities of cucurbitacins from Cucurbita andreana. Cancer Lett..

RETRACTED

[30] Musza L.L., Speight P., McElhiney S., Barrow C.J., Gillum A.M., Cooper R., Killar L.M. (1994). Cucurbitacins, cell adhesion inhibitors from Conobea scoparioides. J. Nat. Prod..

[31] Duncan K.L., Duncan M.D., Alley M.C., Sausville E.A. (1996). Cucurbitacin E-induced disruption of the actin and vimentin cytoskeleton in prostate carcinoma cells. Biochem. Pharmacol..

[32] Kong Y., Chen J., Zhou Z., Xia H., Qiu M.H., Chen C. (2014). Cucurbitacin E induces cell cycle G2/M phase arrest and apoptosis in triple negative breast cancer. PLoS One.

[33] Yang J., Cheng D., Zhou S., Zhu B., Hu T., Yang Q. (2015). Overexpression of X-box binding protein 1 (XBP1) correlates to poor prognosis and up-regulation of PI3K/mTOR in human osteosarcoma. Int. J. Mol. Sci..

[34] Liu Y., Bi T., Dai W., Wang G., Qian L., Shen G., Gao Q. (2015). Lupeol induces apoptosis and cell cycle arrest of human osteosarcoma cells through PI3K/AKT/mTOR pathway. Technol. Cancer Res. Treat..

[35] Jia Q., Cheng W., Yue Y., Hu Y., Zhang J., Pan X., Xu Z., Zhang P. (2015). Cucurbitacin E inhibits TNF-alpha-induced inflammatory cytokine production in human synoviocyte MH7A cells via suppression of PI3K/Akt/NF-kappaB pathways. Int. Immunopharmacol..

